# hPMSC transplantation restoring ovarian function in premature ovarian failure mice is associated with change of Th17/Tc17 and Th17/Treg cell ratios through the PI3K/Akt signal pathway

**DOI:** 10.1186/s13287-018-0772-x

**Published:** 2018-02-14

**Authors:** Na Yin, Yanlin Wang, Xueyan Lu, Ranran Liu, Lianshuang Zhang, Wei Zhao, Wendan Yuan, Qianqian Luo, Hao Wu, Xiying Luan, Hongqin Zhang

**Affiliations:** 1 Department of Histology and Embryology, Binzhou Medical University, 346 Guanhai Rd, Yantai, Shandong China; 2 Reproductive Medicine Center of the Affiliated Hospital of Binzhou Medical College, Binzhou, Shandong China; 3 Reproductive Medicine Center of the Affiliated Hospital of Binzhou Medical College, Yantai, Shandong China; 4 Research Institution of Reproductive Medicine, Binzhou Medical University, Yantai, Shandong China; 5 Basic Medicine College, Binzhou Medical University, Yantai, Shandong China; 6 Department of Morphology Laboratory, Binzhou Medical University, Yantai, Shandong China; 7 Clinical Medical School, Binzhou Medical University, Yantai, Shandong China; 8 Department of Immunology, Binzhou Medical University, 346 Guanhai Rd, Yantai, Shandong China

**Keywords:** Premature ovarian failure, Human placenta-derived mesenchymal stem cells, PI3K, Akt, Immune factors

## Abstract

**Background:**

Human placenta-derived mesenchymal stem cell (hPMSC) transplantation has been demonstrated to be an effective way of recovering ovarian function in mice with autoimmune induced premature ovarian failure (POF). But the exact mechanism remains unclear. The goal of the present study is to investigate the role of immune factors (T-helper 17 (Th17), cytotoxic T (Tc17) and regulatory T (Treg) cells) in the recovery of ovarian function and whether the phosphatidylinositol 3-kinase (PI3K)/Akt signal pathway is involved in the regulation.

**Methods:**

The inhibitor of PI3K/Akt was administered to observe its effect on ovarian function recovery and immune regulation. Serum levels of estradiol (E_2_), follicle stimulation hormone (FSH), luteinizing hormone (LH) and anti-Müllerian hormone (AMH)) and anti-Zona pellucida antibody (AZPAb) were measured by ELISA to evaluate ovarian function. The morphological changes of ovaries were observed by HE staining. Apoptosis of granular cells (GCs) was determined by detecting the expression of capase-3. Expression of p-Akt protein was detected by immunohistochemistry and western blot assay in ovarian tissues. The MTT assay was performed to assess GC proliferation. GC apoptosis was performed using flow cytometry analysis. Percentages of Th17, Tc17 and Treg cells were detected by flow cytometry. Expression of interleukin (IL)-17 in serum was measured by ELISA.

**Results:**

LY294002 administration decreased serum levels of E_2_ and AMH, while the levels of FSH, LH and AZPAb in serum were increased compared with mice in the hPMSC transplantation group. The ovarian morphology presented as atrophy and fibrosis, with functional follicles exhausted. The expression of p-Akt in ovarian tissue was significantly decreased. Also, LY294002 administration significantly decreased proliferation and increased cell apoptosis in GCs, and for immune factors the ratios of Th17/Tc17 and Th17/Treg cells were significantly increased, as well as the serum levels of IL-17.

**Conclusions:**

Our data suggest that the PI3K/Akt signal pathway is involved in the recovery of ovarian function by changing the ratios of Th17/ Tc17 and Th17/Treg cells in POF mice following hPMSC transplantation.

## Background

Premature ovarian failure (POF) is a heterogeneous disorder characterized by the cessation of ovarian function, along with elevated gonadotropins and decreased estrogen levels in women younger than 40 years old [1]. Although the exact causes of POF remain unknown, it is reported that autoimmune mechanisms may be involved in approximately 10–30% of women with POF disorder [2]. Currently, no effective treatment has been found. Many studies are focusing on the potential and alternative therapeutic modality of stem cell therapy, which provides an approach to restore the function of injured tissues [3]. Human placenta-derived mesenchymal stem cells (hPMSCs) are multipotent and nonhematopoietic progenitor cells with high differentiation and proliferation potential, of which the phenotype and characteristics are considered to have great advantages over MSCs isolated from other sources [4]. The recovery of ovarian function following hPMSC transplantation has been demonstrated successfully in our study published previously [5].

The role of the phosphatidylinositol 3-kinase (PI3K)/Akt signal pathway has been widely investigated in cell proliferation, cell transformation, paracrine function and angiogenesis [6–9]. Recent studies have shown that this signal pathway is involved in manipulating the dormancy and activation of mammalian primordial follicles [10, 11]. PI3K stimulates the activation of phosphoinositide-dependent kinases-1/2 (PDK1/2), which then phosphorylate Akt at two critical threonine and serine residues. Phosphorylation of these residues is required for Akt activation [12], as activated Akt phosphorylates various effector molecules. To investigate the mechanisms of how hPMSC transplantation improves ovarian function in POF mice, expression of the PI3K/Akt signaling pathway is investigated in this study.

Additionally, immune regulation is reported to be involved in autoimmune disease progression [13]. For example, T-helper 17 (Th17, CD3^+^CD4^+^IL17^+^T) cells, cytotoxic T (Tc17, CD3^+^CD8^+^IL17^+^T) cells and regulatory T (Treg, CD3^+^CD4^+^CD25^+^Foxp3^+^T) cells are all involved in the pathogenesis of inflammatory and autoimmune diseases. Treg cells secrete immunosuppressive cytokines to suppress the immune response, while Th17 cells can increase the immune response via the release of inflammatory cytokines [14, 15]. The Tc17 subset is a new unique cell lineage, which displays a greatly suppressed cytotoxic function and shares some key features with the Th17 subset [16]. These cells are reported to be involved in inflammation, autoimmune diseases, allergic reactions and infection [17–20]. Since hPMSC transplantation is shown to recover ovarian function in autoimmune-induced POF mice, we investigate whether these immune regulatory cells are involved in the regulation of ovarian function recovery. Furthermore, we investigate whether the regulation is mediated through the PI3K/Akt signal pathway. The data obtained from this study will provide useful information to develop the stem cell therapeutic approach to treat patients with POF in the clinic.

## Methods

### Experimental animals

Six-week-old female (for in-vivo study) and 3-week-old female (for in-vitro study) BALB/c mice were purchased from Jinan Pengyue Experimental Animal Breeding Co., Ltd (Shandong, China). All animals were housed in an animal facility and were fed a standard pellet diet with free access to water. All of the experimental procedures have been approved by the Institutional Animal Care and Use Committee at Binzhou Medical University, and the study was conducted in accordance with the National Research Council Guide for Care and Use of Laboratory Animals.

### Chemicals

The ZP3 peptide was synthesized by an automatic peptide synthesizer (Hangzhou Economic & Technological Development Zone, China), at 91.5% peptide purity as determined by high-performance liquid chromatography (HPLC). The amino acid composition was verified by amino acid analysis and the amino acid sequence of the murine ZP3_330–342_ peptides used in this study was NSSSSQFQIHGPR.

LY294002 (Selleck, USA) was dissolved in DMSO (Sigma, USA) at a stock concentration of 10 mM and added to cell cultures at a final concentration of 0–50 μM.

### Isolation and culture of hPMSCs

hPMSCs were isolated as described in our previous study [21]. Human placentas were collected from pregnant women who were tested negative for HIV-I, hepatitis B and hepatitis C under written and informed consent. This work has been approved by the Institutional Ethics Committee. The placentas were dissected carefully, washed with phosphate-buffered saline (PBS), minced mechanically and digested with 0.1% collagenase IV (Gibco) for 30 min at 37 °C. A 100-μm nylon membrane was used to remove undigested tissue fragments. Cell suspensions were collected and centrifuged at 1500 rpm for 10 min, and the isolated cells were resuspended in low-glucose Dulbecco’s modified Eagle’s Medium (Gibco) supplemented with 10% fetal bovine serum (FBS; Gibco), 100 U/ml streptomycin sulfate and 100 U/ml penicillin G, and were cultured at 37 °C in a humidified atmosphere with 5% CO_2_. To confirm the phenotype of hPMSCs, cell morphology was observed under a light microscope (Olympus, Japan). For osteogenic differentiation, Alizarin Red staining was used to identify osteoblast-like cells. For adipogenic differentiation, Oil Red O staining was used to identify adipose cells. Additionally, the membrane and intracytoplasmic molecular markers of hPMSCs were examined using FCM. After staining with specific hPMSC surface molecule antibody using phycoerythrin-conjugated or fluorescein isothiocyanate-conjugated mouse anti-human CD19, CD73, CD105, CD90, CD34, HLA-DR and CD14 mAb (BD Biosciences and Invitrogen), the cells were sorted with cytometry and harvested for culture [22]. The cells were used for experiment after three passages.

### Isolation, culture and identification of ovarian GCs

Three-week-old female mice were injected intraperitoneally with pregnant mare serum gonadotropin (PMSG; Solarbio) to stimulate follicle growth. Bilateral ovaries were removed under aseptic conditions 48 h later. The adipose and connective tissues of the ovaries were removed and washed with PBS solution, and GCs were isolated under an anatomical microscope and single cell suspensions were obtained. The cells were washed three times and centrifuged at 1000 rpm for 5 min. The GCs were cultured with DMEM/F12 (1:1) medium in 10% fetal bovine serum, streptomycin (100 U/ml; Gibco), penicillin (100 U/ml; Gibco) and FSH (50 ng/ml; Solarbio) at 37 °C in a humidified atmosphere with 5% CO_2_. The first passage of GCs was used in all experiments.

The follicle stimulating hormone receptor (FSHR) of the GCs was assessed by immunofluorescent. Briefly, after 4% paraformaldehyde fixation and 0.1% Triton X-100 penetrating cell membrane, GCs were incubated overnight at 4 °C with rabbit anti-mouse FSHR antibody (dilution 1:150). After washing in PBS, the cells were incubated for 1 h at 37 °C with a secondary biotinylated donkey anti-rabbit IgG antibody (dilution 1:300). The cells were then washed in PBS and incubated for 10 min at 37 °C with DAPI dye liquor. The staining of FSHR was recorded with a laser confocal microscope (Olympus CKX41).

### Animal model establishment

Adult mice (*n* = 60) were divided randomly into five groups (*n* = 12 each): control group (C group), POF group (M group), POF + hPMSCs group (T group), POF + hPMSCs + LY294002 group (L group) and POF + hPMSCs + DMSO group (D group). Groups M, T, L and D were first injected subcutaneously with 50 nmol/L of ZP3 (mouse) emulsified in complete Freund’s adjuvant (CFA) (*Mycobacterium tuberculosis* H37RA strain, 0.16 mg/mouse; Sigma) 1 week after adaptive feeding, and then injected with 50 nmol/L of ZP3 (mouse) emulsified in Freund’s incomplete adjuvant (FIA) (*M. tuberculosis* H37RA strain, 0.16 mg/mouse; Sigma) 2 weeks later. Mice in group C received no treatments. The cell suspension containing 1 × 10^6^ hPMSCs of the sixth passage were injected into mice in groups T, L and D after 1 week, according to the studies published previously [23, 24]. PBS was injected into mice in group M as vehicle control. One week later, mice in group L were treated with 1 mg LY294002 dissolved in DMSO plus 0.25 ml of PBS with daily IP injection for 3 weeks. The selection of this dose is based upon a preliminary dose-ranging study from 0–100 mg/kg body weight of LY294002 (i.p.) in which 100 mg/kg was found to result in significant inhibition of ascites and tumor burden [25]. Mice in group D were treated with DMSO vehicle control via IP injection. The concentration of DMSO in vehicle control was 8%. At day 21, all mice were sacrificed to evaluate the effect of LY294002 on restoring function following hPMSC transplantation into mice with POF.

### Hormone (E_2_, FSH, LH, AMH), AZPAb and IL-17 measurement in serum

Blood samples were obtained from postcava and centrifuged at 4000 rpm for 10 min. The serum levels of estradiol (E_2_), follicle stimulation hormone (FSH), luteinizing hormone (LH), anti-Müllerian hormone (AMH), anti-Zona pellucida antibody (AZPAb) and IL-17 concentration were measured by ELISA kits (Mlbio, China) according to the manufacturer’s instructions.

### Ovarian follicle counting and morphological analysis

The ovarian tissues were collected, fixed and stained for histopathological examination using light microscopy (Olympus). The follicles were counted only on those containing an oocyte with a clearly visible nucleus. The follicles were categorized as primordial, primary, secondary and atretic follicles, according to the method described previously [26].

### Immunohistochemistry

Ovaries from treated and control mice were fixed and cut into sections (4 μm), and then incubated with rabbit primary polyclonal antibodies against mouse cleaved PI3K (1:100 dilution; Proteintech) and Capase-3 (1:100 dilution; Proteintech), Akt (Ser 473, 1:200 dilution; Proteintech) and p-Akt (1:200 dilution; Proteintech) at 4 °C overnight. After that, incubation with biotinylated secondary antibodies was conducted at 37 °C for 30 min. The reaction products were developed with diaminobenzidine (DAB) as chromogen and counterstained with hematoxylin. The staining results were scored using the German immunoreactive score (IRS). The staining intensity was graded as “0” (negative), “1” (weak), “2” (moderate) and “3” (strong); staining extent was graded as “0” (<5%), “1” (5–25%), “2” (25–50%), “3” (50–75%) or “4” (> 75%). Values of the staining intensity and the staining extent were multiplied as a final IRS [27].

### Western blotting analysis

For western blotting analysis, ovaries were lysed using radioimmunoprecipitation assay (RIPA) buffer and the protein concentration was measured by bicinchoninic acid assay. Proteins were separated using 10% sodium dodecyl sulfate polyacrylamide gel electrophoresis (SDS-PAGE) and transferred to a polyvinylidene difluoride (PVDF) membrane. The membrane was blocked with 6% milk powder at room temperature, followed by addition of primary antibodies against Akt (1:1000; Proteintech), p-Akt (1:1000; Proteintech) and GAPDH (1:50,000; Proteintech) for overnight incubation at 4 °C on a shaking table. The membrane was then washed three times, and incubated with secondary antibodies for 1 h at room temperature. Protein expression was detected using the Super Enhancer chemiluminescence (ECL) Kit (Novland, China), and band intensity was quantified using ImageJ software.

### Determination of cell viability by MTT assay

The effect of LY294002 on GC viability with or without hPMSC supernatant coculture was determined by 3-(4,5-dimethylthiazoyl-2-yl)2,5-diphenyltetrazolium bromide (MTT) assay. Briefly, cells were seeded at a density of 2000 cells/scaffold and cocultured with supernatant of hPMSCs (0–100 μl) in 96-well plates, and maintained at 37 °C under 5% CO_2_ for 24 h. The medium was then added with LY294002 (0–50 μm) for an additional 24, 48 or 72 h. The concentration of DMSO in both control and test groups was maintained at 0.5%. The culture medium of each cultured specimen was removed, and 20 μl of MTT solution (0.5 mg/ml) was added to each well. After incubation for 4 h, the MTT solution was removed. The formazan crystals were dissolved in 150 μl DMSO and the plate was kept at room temperature in dark place for 10 min on a rotary shaker. The absorbance of plates was measured at 490 nm with a plate reader (Infinite 200 Pro; Tecan, Switzerland).

### Apoptosis assay by FCM

Apoptotic GCs were assessed using the FITC Annexin V apoptosis detection kit (BD Pharmingen, USA). GCs were collected, washed three times with PBS and resuspended in 500 μl of cold 1× binding buffer, mixed with 5 μl of Annexin-V-fluorescein isothiocyanate (FITC) and 5 μl of propidium iodide (PI), and eventually detected using FCM (FACSVantage diva, USA).

### Differentiation of T-lymphocyte subset by FCM

To determine the ratios of Th17/Treg and Th17/Tc17 cells in mice, FCM analysis was performed on isolated spleen cells using anti-mouse CD3, CD4, CD8, CD25, IL-17 and Foxp3 monoclonal antibodies. The spleens were minced mechanically and lysed in lymphocyte separation medium. The isolated spleen cells were washed and resuspended in PBS. Anti-mouse CD3 APC, Anti-mouse CD4 FITC and Anti-mouse CD25 Percp-cy5.5/Anti-mouse CD8 Percp-cy5.5 (eBioscience, San Diego, USA) were then mixed at 4 °C for 10 min in the dark. After cell membranes were ruptured, Anti-mouse Foxp3 PE/Anti-mouse IL-17 PE (eBioscience) was added to the cell suspension and analyzed using FCM.

### Data analysis

Analyses were performed using SPSS 16.0 software. Each experiment was performed at least three times, and the experimental continuous data are shown as the mean ± standard deviation. Results were analyzed statistically using Student’s *t* test for comparisons between two groups. A one-way analysis of variance (ANOVA) was used to the distribution of data. *P* < 0.05 was considered statistically significant.

## Results

### hPMSC phenotype characterization

The cells isolated from human placenta began to form individual clone spheres after 7–10 days of inoculation and show fibroblast-like morphology (Fig. 1b). The adherent cells can be expanded in easily vitro by several cycles of trypsinization. A homogeneous cell population was observed after three passages. Even following 10 passages, the cells still retain the same morphology without any changes. Immunophenotyping analysis showed the positive expression of mesenchymal progenitor markers with CD73, CD90 and CD105. The hematopoietic cell surface markers CD14, CD34 CD19 and HLA-DR are shown as negative (Fig. 1a). In an ex-vivo conditional culture system, hPMSCs were induced to develop into different lineages. In osteoblastic induction medium, Alizarin Red staining showed calcium deposition (Fig. 1c). In adipogenic induction medium, fat globules were present in the cytoplasm, and Oil Red O staining was positive (Fig. 1d). These results are consistent with the previous literature reports and confirm the phenotype of hPMSCs [22].

**Fig. 1:** Cell surface markers, morphology and pluripotency of hPMSCs and GCs. Green histograms represent isotype control staining; blue histograms represent expression of indicated cell surface marker (**a**). hPMSCs cultured under conditions for differentiation into osteoblasts or adipogenesis (**b**–**d**). Cultured hPMSCs shows fibroblast-like morphology (**b**, ×200). Osteoblasts are displayed by Alizarin Red staining; darker red staining indicates calcium deposition (**c**, ×200). Adipogenesis displayed by accumulation of neutral lipid vacuoles stained with Oil Red O (**d**, ×200). Morphology and phenotypes of GCs (**e**–**h**). GCs shown as spindle-shaped morphology (**e**, ×200). DAPI staining (blue fluorescence) indicates the GC nucleus (**f**, ×400). FSHR-positive expression identified under Dylight 549 (red fluorescence) (**g**, ×400). Double-labeled staining (blue and red fluorescence) cells defined as FSHR-positive expression in GCs (**h**, ×400). FITC Annexin-V-fluorescein isothiocyanate, PE phycoerythrin

### GC identification

The GCs were isolated and cultured as a monolayer. The cells were observed as polygonal or cuboidal morphologic characteristics, under inverted phase-contrast microscopy (Fig. 1e). Immunofluorescence staining with FSHR antibody was used as a marker to identify the GCs. The data showed most cells within FSHR-positive staining, which was localized in the cytoplasm (Fig.1f–h).

### E_2_, FSH, LH, AMH, AZPAb and IL-17 levels in serum

We investigated the effect of LY294002 on hormone (E_2_, FSH, LH, AMH), AZPAb and IL-17 secretion in serum of POF mice after hPMSC transplantation. The results in Fig. 2 show that the serum levels of E_2_ and AMH were significantly decreased, while the levels of FSH, LH and AZPAb were increased in POF mice compared to the control group (*P* < 0.001). Serum levels of E_2_ and AMH are increased, along with decreased levels of FSH, LH and AZPAb (*P* < 0.001) following hPMSC transplantation. After LY294002 treatment, the increased E_2_ and AMH levels were reduced; however, the serum levels of FSH, LH, AZPAb were increased (*P* < 0.001). Additionally, hPMSC transplantation significantly decreased the production of IL-17 compared with POF mice without hPMSC transplantation (*P* < 0.001). Following LY294002 treatment, this trend was reversed with increased levels of IL-17 (*P* < 0.01). Based upon these results, it can be concluded that the PI3K/Akt signal pathway is involved in ovarian function recovery in POF mice following hPMSC transplantation.

**Fig. 2:** Effects of LY294002 on the serum levels of E_2_, FSH, LH, AMH, AZPAb and IL-17 in POF mice with or without hPMSC transplantation. **a** Estradiol (E_2_) release. **b** Follicle stimulation hormone (FSH) release. **c** Luteinizing hormone (LH) release. **d** Anti-Müllerian hormone (AMH) release. **e** Anti-Zona pellucida antibody (AZPAb) release. **f** Interleukin (IL)-17 release. Data presented as mean ± SD. ^**^P < 0.01, ^***^P < 0.001 vs POF group. Groups: C control, M POF, T POF + hPMSCs, L POF + hPMSCs + LY294002, D POF + hPMSCs + DMSO. POF premature ovarian failure, hPMSC human placenta-derive mesenchymal stem cell, DMSO dimethylsulfoxide

### Histological examination and follicle count

In the negative control group, the ovary contains a large number of healthy follicles at all stages, including primordial follicles (Fig. 3A-a), primary follicles (Fig. 3A-b), secondary follicles (Fig. 3A-c) and atretic follicles (Fig. 3A-d). In contrast, the ovaries of mice in the POF group and the POF + hPMSCs + LY294002 group showed atrophied ovaries composed of interstitial cells in a fibrous matrix, with a reduced number of follicles at each stage of development (Fig. 3B, D). The number of functional follicles (primordial follicles, primary follicles and secondary follicles) in POF mice were significantly decreased compared to the control group (*P* < 0.001). After hPMSC transplantation, the number of healthy follicles was significantly increased (*P* < 0.05). After LY294002 treatment, the number of healthy follicles showed a declined trend (*P* < 0.05) and there is no statistical difference with the POF group (*P* > 0.05).

**Fig. 3:** Histopathological examination of ovarian tissues. Photomicrographs (100×) show hematoxylin and eosin stained ovaries. (**A**) Control group (C group); four types of ovarian follicles observed (a–d). (**B**) POF group (M group). (**C**) POF + hPMSCs group (T group). (**D**) POF + hPMSCs + LY294002 group (L group). (**E**) POF + hPMSCs + DMSO group (D group). (**F**) Quantitation on follicle count from ovaries in mice of the five groups. Data presented as mean ± SD. ^*^P < 0.05, ^**^P < 0.01, ^***^P < 0.001 vs POF group. Bar scale = 200 μm. POF premature ovarian failure, hPMSC human placenta-derive mesenchymal stem cell, DMSO dimethylsulfoxide

### PI3K, Akt, p-Akt and capase-3 expression in ovarian tissues

Immunohistochemistry (IHC) was used to measure the expression of PI3K, Akt, p-Akt and capase-3 in ovarian tissues of all group mice. All of these signals were mainly localized in the cytoplasm (Fig. 4). Expression of PI3K and Akt was observed in the ovarian tissues without significant differences among each group (*P* > 0.05) (Fig. 4a, b). Expression of p-Akt in POF mice was lower than in the control group (*P* < 0.01). After hPMSC transplantation, p-Akt protein expression was greatly increased (*P* < 0.01). With the administration of LY294002, positive staining for p-Akt protein was decreased (*P* < 0.01) (Fig. 4c). Expression of capase-3 protein was higher in POF mice compared to the POF mice with hPMSC transplantation (*P* < 0.01). However, after LY294002 treatment, caspase-3 expression was increased (*P* < 0.01) (Fig. 4d). These results indicate that the PI3K/Akt signal pathway is involved in the recovery of ovarian function induced by hPMSC transplantation in POF mice.

**Fig. 4:** IHC analysis on PI3K, Akt, p-Akt and capase-3 in ovarian tissue of mice. Photomicrographs (400×) show hematoxylin and DAB-stained ovaries. (**a1-d1**) Control group (C group). (**a2-d2**) POF group (M group). (**a3-d3**) POF + hPMSCs group (T group). (**a4-d4**) POF + hPMSCs + LY294002 group (L group). (**a5-d5**) POF + hPMSCs + DMSO group (D group). The statistical charts of the four kinds of cytokines expression in the five groups (**a6**-**d6**). Brown in cytoplasm indicates positive expression of the aimed protein. Blue represents cell nuclear staining. ^**^P < 0.01, ^***^P < 0.001 vs POF group. Bar scale = 50 μm. POF premature ovarian failure, hPMSC human placenta-derive mesenchymal stem cell, DMSO dimethylsulfoxide, PI3K phosphatidylinositol 3-kinase

### AKT activation by western blot analysis

To determine whether Akt is involved in the recovery of ovarian function in POF mice after hPMSC transplantation, western blot analysis was performed to analyze the phosphotransferase activity of Akt protein. GAPDH was used as an internal control (Fig. 5a). AKT protein showed no difference in the five groups (*P*>0.05)(Fig. 5b). In the POF + hPMSCs group, the kinase activity of Akt was increased compared to the POF group (*P* < 0.05), which suggests that the PI3K/Akt signal pathway was activated. When treating the mice with LY294002, expression of p-Akt was significantly decreased (*P* < 0.05) (Fig. 5c). These findings further support that the PI3K/Akt pathway is involved in the recovery of ovarian function in POF mice after hPMSC transplantation.

**Fig. 5:** AKT expression in ovarian tissues by western blot analysis. Akt and p-Akt protein expression (**a**) and quantification of Akt (**b**) and p-Akt (**c**) protein expression. Values expressed as mean ± SD. ^**^P < 0.01, ^***^P < 0.001 vs POF group. Groups: C control, M POF, T POF + hPMSCs, L POF + hPMSCs + LY294002, D POF + hPMSCs + DMSO. POF premature ovarian failure, hPMSC human placenta-derive mesenchymal stem cell, DMSO dimethylsulfoxide

### Effects of LY294002 on proliferation of GCs when cocultured with or without the supernatant of hPMSCs

To analyze the effect of inhibiting the PI3K/Akt signal pathway on GC proliferation, the cells were treated with different concentrations of PI3K inhibitor LY294002 in the presence or absence of hPMSCs. Considering hPMSCs and GCs are both anchorage-dependent cells and have similarity in morphology, the supernatant of hPMSCs with a large amount of cytokines produced was used for further study. As determined by the MTT assay, the cell viability was significantly decreased in the group of GCs cocultured with 50 μl supernatant of hPMSCs at 48 and 72 h compared with that measured at 24 h (*P* < 0.05), and the downtrend was slowed at 72 h compared with 48 h (Fig 6a). The effect may be induced by the cytokines produced by hPMSCs, which stimulated the growth of GCs. When cocultured with 100 μl supernatant, GC proliferation was mostly decreased at 48 h (*P* < 0.05) (Fig 6b). The results demonstrated a dose-dependent effect of LY294002 on the inhibition of GC proliferation at the concentrations of 0, 10, 20 and 50 μM when cocultured with the supernatant of hPMSCs (50 or 100 μl) for 24, 48 and 72 h (Fig. 6c, d). These results suggest that LY294002 exhibits antiproliferative effects on GC cell growth.

**Fig. 6:** Effect of LY294002 on GC proliferation and apoptosis when cocultured with the supernatant of hPMSCs. The tendency charts of GC proliferation cocultured with 50 μl (**a**) or 100 μl (**b**) supernatant of hPMSCs. The statistical charts of GC proliferation cocultured with 50 μl (**c**) or 100 μl (**d**) supernatant of hPMSCs. **e** Representative flow cytometric plot for GCs apoptosis in different condition, and the percentage of cells in the upper right quadrant indicates late apoptotic cells. **f** The statistical chart of GCs apoptosis in all groups. Values expressed as mean ± SD. ^*^P < 0.05, ^**^P < 0.01, ^***^P < 0.001 vs POF group. GC granular cell, hPMSC human placenta-derive mesenchymal stem cell, DMSO dimethylsulfoxide, FITC Annexin-V-fluorescein isothiocyanate, PE phycoerythrin, OD optical density

### Effects of GC apoptosis with LY294002 treatment

To elucidate the effect of LY294002 on GC apoptosis in POF mice with hPMSC transplantation, FCM analysis was performed. A total 100 μl of supernatant of hPMSCs was used in this analysis, and the cellular apoptosis was measured after 24 h of culture. The dose–response effect of LY294002 on GC apoptosis when cocultured with the supernatant of hPMSCs was evaluated. Results show that when GCs were treated with LY294002 (0–50 μM) in the presence of the supernatant of hPMSCs for 24 h, the percentage of apoptotic bodies in GCs was increased to 10.14%, 18%, 18.05% and 20.24%, respectively (Fig. 6). LY294002 (0–50 μM) significantly decreased the population of GCs in a concentration-dependent manner.

### Effects of LY294002 on hPMSC transplantation induced Th17/Tc17 ratio and Th17/Treg cells in POF mice

To determine whether hPMSC transplantation changes the ratios of Th17/Tc17 and Th17/Treg cells during the recovery of ovarian function in POF mice, T cells were harvested from spleens and Th17, Tc17 and Treg cells were isolated and sorted by FCM (Fig. 7a, b,c). As shown in Fig. 7d, the percentage of Th17 cells was upregulated in the POF group compared with that in the control group (*P* < 0.01). Following hPMSC transplantation, the increased Th17 cells reduced, and this tendency was reversed after LY294002 treatment (*P* < 0.05). The percentage of Treg cells showed an opposite tendency, which was declined in POF mice (*P* < 0.001), and then increased after hPMSC transplantation (*P* < 0.01) but declined with LY204002 administration (*P* < 0.01) (Fig.7f). The ratios of Th17/Tc17 (Fig. 7e) and Th17/Treg (Fig. 7g) cells significantly increased in the POF group compared to the control group (*P* < 0.001). Following the hPMSC transplantation, the ratios were significantly decreased (*P* < 0.05). With LY294002 treatment, the ratios increased again (*P* < 0.01). These data suggest that LY294002 is involved in the immune regulation on the recovery of ovarian function in POF mice following hPMSC transplantation.

**Fig. 7:** Effects of LY294002 on ratios of Th17/Tc17 and Th17/Treg cells. (**a–c**) Representative flow cytometric plots for Th17, Tc17 and Treg cell subset acquisition isolated from spleens, respectively. **d** Th17 cell population comparison among the groups. **e** Ratios of Th17/Tc17 comparison among the groups. **f** Treg cell population comparison among the groups. **g** Ratios of Th17/Treg comparison among the groups. Data expressed as mean ± SD. ^*^P < 0.05, ^**^P < 0.01, ^***^P < 0.001 vs POF group. Groups: C control, M POF, T POF + hPMSCs, L POF + hPMSCs + LY294002, D POF + hPMSCs + DMSO. POF premature ovarian failure, hPMSC human placenta-derive mesenchymal stem cell, DMSO dimethylsulfoxide, FITC Annexin-V-fluorescein isothiocyanate, PE phycoerythrin, IL interleukin

## Discussion

Increasing numbers of reports suggest that stem cell transplantation is a promising treatment for POF [28–31]. hPMSC transplantation has been recognized as an ideal source for clinical applications to treat diseases due to its easy accessibility, high differentiation and proliferation potential and low immunogenicity [32]. Especially, hPMSCs have immunosuppressive features with low expression of MHC I but not MHC II antigens [33], giving them an advantage for transplantation as they have almost no allograft reactions. However, the transplantation of hPMSCs faces some challenges and limitations. For example, the optimal time window for collection and culture, the preservation, the dosage, the route and frequency of hPMSC administration, the safety of post transplantation and the long-term survival rates still need to be investigated [31]. The goal of this study is to investigate whether the PI3K/Akt signal pathway is involved in the ovarian function recovery in POF mice after hPMSC transplantation, and its regulation on immune factors (Th17, Tc17 and Treg cells). The study was conducted on a successfully established POF mice model with ZP3 treatment. The inhibitor of the PI3K/Akt signal pathway was administered in POF mice with or without hPMSC transplantation to investigate its role in the recovery of ovarian function.

To evaluate ovarian function, the serum levels of AMH, AZPAb, E_2_, FSH and LH were measured. AMH is involved in regulation of folliculogenesis and is considered the best predictor of ovarian reserve [34]. The presence of AZPAb in serum is reported to be associated with ovarian dysfunction, and induces infertility by interfering with the sperm–oocyte interaction in women [35]. The elevated serum levels of AMH and E_2_ and decreased FSH, LH and AZPAb in mice receiving hPMSC transplantation demonstrate the successful recovery of ovarian function in mice with ovarian failure. Additionally, it is observed that hPMSC transplantation can significantly increase the functional follicle numbers. Also, lower positive expression levels of capase-3 were detected, which represents a significant decrease of apoptotic GCs and can result in an increase in healthy oocyte GCs to facilitate the recovery of ovarian function in POF mice [36]. All of these findings suggest that hPMSC transplantation successfully restores ovarian function in POF mice.

It is reported that the PI3K/Akt signal pathway plays an important role in folliculogenesis [37], and also controls the survival, loss and activation of primordial follicles in the oocyte [38, 39]. Additionally, recent studies show that this pathway plays a critical role in immunity and autoimmunity [40]. However, it is unclear whether this signal pathway is associated with the repairing process of autoimmune-induced ovarian failure in POF mice receiving hPMSC transplantation. In this study, we used a PI3K/Akt signal pathway inhibitor LY294002 to determine the mechanism of ovarian function recovery. Our data show that LY294002 demonstrated a remarkable growth-inhibitory and apoptosis-inducing effect in the GCs cocultured with the supernatant of hPMSCs in vitro*.* Also, decreased expression of p-Akt was detected in the ovarian tissues. Compared with those mice receiving hPMSC transplantation only, the inhibitor caused decreased levels of AMH and E_2_ but increased levels of FSH, LH and AZPAb in the serum of mice with LY294002 treatment when compared with POF mice with hPMSC transplantation only; HE staining revealed an apparent shrinkage of functional follicle number and a lower percentage of apoptotic GCs after blocking the PI3K/Akt pathway. These results indicated the PI3K/Akt signal served an important role in the recovery of ovarian function in mice with hPMSC transplantation.

Th17 and Tc17 cells are known play an important pathogenic role in several models of autoimmune diseases [41]. In the present study, we also investigated whether these immune cells are involved in the regulation of ovarian function recovery following hPMSC transplantation in POF mice. Also, the PI3K/Akt inhibitor was administered to determine whether this signal pathway was involved in the immune regulation. After LY294002 treatment, the data showed that only the percentage of Th17 cells was significantly increased but not that of Tc17 cells. Also, the Th17/Tc17 cell ratio significantly increased in mice after LY294002 treatment. Since Th17 cells and Tc17 cells are characterized by the production of IL-17, it is observed that significantly higher expression of serum IL-17 levels in the POF + hPMSCs + LY294002 group further support these results. Additionally, Treg cells play an important role in suppressing host immunity [42], and the immune suppression function can be converted into inflammatory cytokine-producing cells in a specific inflammatory microenvironment, gradually lose Foxp3 expression and finally transdifferentiate into Th17 cells, which potentially contribute to disease pathogenesis [43, 44]. The decreased Treg cells most likely lead to low tolerance of autoimmunity and result in the progression of POF disease. In addition to the decrease of Treg cells, an imbalance between Th17 and Treg cells was also found in the POF group. The administration of LY294002 affects the ratio of Th17 and Treg cells in POF mice. The Treg cells most likely counteract Th17 cells to maintain the immune balance in a normal condition. The changes in the Th17/Treg and Th17/Tc17 cell ratios indicate the association of host immunity and POF disease. hPMSC implantation may affect these immune cells and promote the recovery of ovarian function. During this process, the PI3K/Akt signal pathway is involved in this regulation.

## Conclusions

We have shown that hPMSC transplantation can lead to recovery of injured ovarian function induced by ZP3 immunization in mice. The restoring function is associated with the PI3K/Akt signal pathway, and the balance between the ratios of Th17/Tc17 and Th17/Treg cells. These findings may provide useful information to further investigate the mechanism of ovarian function recovery in POF mice following hPMSC transplantation.

## Abbreviations

AMH: Anti-Müllerian hormone
AZPAb: Anti-Zona pellucida antibody
GC: Granular cell
CFA: Complete Freund’s adjuvant
E_2_: Estradiol
FBS: Fetal bovine serum
FCM: Flow cytometry
FITC: Annexin-V-fluorescein isothiocyanate
FSH: Follicle stimulation hormone
FSHR: Follicle stimulating hormone receptor
hPMSC: Human placenta-derive mesenchymal stem cell
IFA: Freund’s incomplete adjuvant
IHC: Immunohistochemistry
LH: Luteinizing hormone
MTT: 3-(4,5-Dimethylthiazoyl-2-yl)2,5-diphenyltetrazolium bromide
PBS: Phosphate-buffered saline
PDK1/2: Phosphoinositide-dependent kinases-1/2
PI3K: Phosphatidylinositol 3-kinase
RIPA: Radioimmunoprecipitation assay
POF: Premature ovarian failure
PVDF: Polyvinylidene difluoride
SDS-PAGE: Sodium dodecyl sulfate polyacrylamide gel electrophoresis
